The article "A Meta-Analysis of the Efficacy of Albumin Paclitaxel versus Docetaxel in the Treatment of Breast Cancer" was retracted in 2023. Reasons: signs of a paper mill; suspected computer-generated content; unreliable results or conclusions; concerns about the data.

# A Meta-Analysis of the Efficacy of Albumin Paclitaxel versus Docetaxel in the Treatment of Breast Cancer

**DOI:** 10.1155/2021/7020177

**Published:** 2021-12-08

**Authors:** Huixin Xu, Yue Li, Jianming Guo, Yuan Sui, Baihui Chen, Dalin Li, Jiakang Jiang

**Affiliations:** ^1^Heilongjiang University of Chinese Medicine, Harbin, China; ^2^Harbin Medical University Cancer Hospital, Harbin, China

## Abstract

**Objective:**

To use meta-analysis to systematically compare the efficacy and adverse reaction rates of albumin paclitaxel and docetaxel in the treatment of breast cancer.

**Methods:**

This study included Chinese and English literature studies on clinical controlled studies of albumin paclitaxel and docetaxel in the treatment of breast cancer by searching CNKI, Weipu, Wanfang, PubMed, Embase, and Cochrane Library. Two researchers participated in the screening of the literature, used the inclusion and exclusion criteria as reference indicators, extracted relevant data, and used the software RevMan5.3 to conduct quality evaluation and meta-analysis of the literature.

**Results:**

4 literature stuides were retrieved that met the inclusion criteria, with 243 study subjects. The included literature had a lower risk of bias. Meta-analysis results showed that compared with the docetaxel group, the protein paclitaxel group had significant differences in objective effective rate (ORR) (OR = 1.56, 95% CI (0.80, 3.03), *P*=0.19), complete remission (CR) (OR = 1.79, 95% CI (0.96, 3.35), *P*=0.07), partial remission (PR) (OR = 0.88, 95% CI (0.53, 1.47), *P*=0.62), nausea (OR = 0.87, 95% CI (0.51, 1.74), *P*=0.84), and vomiting (OR = 0.62, 95% CI (0.45, 1.78) *P*=0.76). The reason may be that the number of literatures included in this study is small or the sample size is insufficient. However, it had an advantage in the incidence of neutropenia (OR = 0.38, 95% CI (0.16, 0.88), *P*=0.02), and the difference between the two groups was statistically significant.

**Conclusion:**

Albumin paclitaxel treatment can better reduce the incidence of neutropenia in breast cancer patients and is of great significance to the safety of breast cancer patients.

## 1. Introduction

Breast cancer is a highly heterogeneous disease. The main reason for its occurrence is the mutation of HER2, BRCA1, BRCA2, RB, and other genes in patients due to factors such as heredity, environment, age, lifestyle, and diet. Paclitaxel is a broad-spectrum anticancer drug extracted from *Taxus brevifolia* and has shown good clinical efficacy in breast cancer tumors [1]. Albumin-bound paclitaxel is a new type of cytotoxic drug that binds to human albumin to form 130 nm-sized particles. The albumin part can bind to the albumin surface receptor on the surface of the vascular endothelial cell membrane to bind paclitaxel. Transported to tumor tissue through endocytosis can have higher antitumor response, prolong tumor progression time, and lower allergic reactions [2]. Docetaxel is a cytotoxic taxane compound obtained by semisynthesis of noncytotoxic precursor compounds extracted from European yew [3]. It has good anticancer activity and is widely used chemotherapy for breast cancer. Albumin paclitaxel and docetaxel are widely used in the treatment of breast cancer, but few people have compared their efficacy and safety in the treatment of breast cancer. Based on this, this study will adopt the method of meta-analysis and search foreign literature databases. A comprehensive and systematic comparison of the clinical efficacy and safety of albumin paclitaxel and docetaxel in the treatment of breast cancer provides ideas for the treatment of breast cancer of paclitaxel drugs.

## 2. Materials and Methods

### 2.1. Search Method

We searched PubMed, Science Net, Science Direct, China Knowledge Network (CNKI), Google Scholar, and other databases. The limited time for searching documents is from the establishment of the abovementioned database to September 2021. The search keyword mainly included “Albumin paclitaxel,” “docetaxel,” “breast cancer,” “breast cancer neutrophils,” and “chemotherapy for breast cancer,” and the search method is Boolean logic search and exact phrase or phrase search. At the same time, in order to avoid missing or missing related documents, screening is also required. The references in the literature were searched for a second time, and the references were read and checked one by one, and the documents related to this research were selected.

### 2.2. Inclusion and Exclusion Criteria

#### 2.2.1. Inclusion Criteria

(1) Literature source: Chinese and English literature on controlled trials of albumin paclitaxel versus docetaxel in the treatment of breast cancer published by major databases. (2) Research objects: patients who were diagnosed with breast cancer by clinical pathological examination and had no previous mental illness or disturbance of consciousness; exclude patients with other malignant tumors. (3) Intervention measures: the test group was given paclitaxel albumin, and the control group was given docetaxel.

#### 2.2.2. Exclusion Criteria

(1) Documents published repeatedly in the same research; (2) conference-published papers, reviews, and documents with incomplete basic data; (3) documents with no full-text data but only abstracts; (4) retrospective research documents; (5) the literature on the measurement indicators of this study has not been evaluated.

### 2.3. Outcome Indicators

Analysis of postoperative indicators of breast cancer patients in the experimental group and the control group: objective response rate (ORR), complete remission (CR), partial remission (PR), neutropenia, nausea, and vomiting.

### 2.4. Document Screening and Data Extraction

Two researchers participated in the screening of the literature, their reference criteria were the inclusion and exclusion criteria, and they worked independently. The first round of work is to delete the duplicated documents from various databases, and then they read the abstract part and all of the documents in a deeper level, and they removed the documents and articles in which the original text cannot be completely obtained. The documents with incomplete results of the experiment are removed. If there are differences between the two participants when solving these problems, then it is necessary to find the original text again, and the researcher reanalyzes and discusses the original text. If the two researchers are still unable to agree, then a third person needs to be found to participate in this discussion.

Researchers used standard data extraction methods when extracting data. The extracted content includes (1) The title of the article, the name of the author, the time the article was published, and the name of the research center; (2) the treatment plan of the experimental group and the control group; (3) the type of malignant tumor that the patient suffered and the basic personal information of the patient at the time; (4) the indicators of the selected study outcome, including ORR, CR, PR, and after the patient's medication. Various adverse reactions occurred, including nausea, vomiting, hair loss, neutropenia, and other events.

### 2.5. Literature Quality Evaluation and Bias Risk Evaluation

When evaluating the quality of the article, the two participating researchers evaluated independently. If there is a conflict between the two parties, and if there are opposite opinions, they can ask the opinions of the third party and then discuss further. Finally, the two participating researchers got the same result. When evaluating the quality of the selected articles, the two participants must strictly follow certain standards, which are the standards of the Cochrane 5.3 manual, and give “A low risk,” “B unclear,” and “C High-risk” results. Before the evaluation, we must first understand the source of bias in the literature results. There are the following aspects: (1) in the process of conducting the experiment, did the experimenters make correct random allocation; (2) if there is correct random allocation, is there any reasonable effective hiding of doctors and patients, and can they estimate the allocation plan; (3) have the doctors and patients been blinded; (4) is the data about the results in the article complete, yes/no/missing; (5) did the researchers report the data completely when they made the final report; (6) whether there were any other sources of bias [4–7].

### 2.6. Statistical Analysis

When we conduct metasystem analysis on the extracted data, we need to learn to use the relevant software, RevMan5.3. There is a value of *I*^2^ in the analysis. Its function is to judge whether there is heterogeneity. If *I*^2^ > 50% and *P* value <0.1, then there is heterogeneity in these data, then we have to check whether the extracted data is accurate and whether the method used is correct when extracting. If there is no error, then we need to adopt a random effects model; if the result shows that *I*^2^ < 50% and *P* value >0.1, then it can be determined that there is no heterogeneity in these data, which means that we can directly use the fixed-effects model. In the process of meta-analysis, various types of bias will appear, and the funnel chart is a good tool for discovering various biases. It has the advantage of intuitiveness.

## 3. Results

### 3.1. Document Screening Process and Results

In this study, we searched a total of 486 articles, and then after the first round of screening, we screened out the repeated articles in various databases. In this process, we screen out 145 articles, and then we screen out 283 articles, including those that have no obvious relationship with the research content and without a complete article. The types of articles are review and case reports. Then, we read all the articles in a deeper level and deleted a total of 54 articles, including those with incomplete experimental data. Finally, we selected a total of four documents for this study and then extracted the data in these four articles for summary and then performed the final meta-analysis. The specific screening process details are shown in Figure 1.

### 3.2. Basic Characteristics and Risk Bias Assessment of Included Studies

Among the four literatures included in this study, three literatures did not mention random double-blind [8–10], and one literature mentioned random double-blind [11]. A total of 243 patients were included in the four articles. The experimental group was albumin paclitaxel, and the control group was docetaxel or docetaxel combined with other drugs, as shown in Table 1. The quality evaluation and bias evaluation of these four articles were carried out in strict accordance with the standards of the Cochrane 5.3 manual. The results are shown in Figures 2 and 3.

### 3.3. Meta-Analysis Results

#### 3.3.1. Objective Efficiency (OR)

In this study, four articles reported two paclitaxel ORR in treatment of breast cancer patients, and extracted data, using RevMan5.3 software to test their heterogeneity, as shown in Figure 4 (*P*=0.83, *I*^2^ = 0%), so there is no heterogeneity between these studies. Then, a fixed effect model was used to carry out meta-analysis of these data and the combined effect (OR = 1.56, 95% CI (0.80, 3.03)). The results showed that the ORR of the paclitaxel group was higher than that of the docetaxel group (*Z* = 1.31, *P*=0.19), which indicated that the difference was not statistically significant. This result suggested that there was no significant difference in the treatment of ORR between the paclitaxel group and the albumin paclitaxel group.

#### 3.3.2. Complete Response Rate (CR)

The four articles in this study all reported the CR of two types of paclitaxel in breast cancer patients. The data were extracted, and RevMan5.3 software was used to test the heterogeneity, as shown in Figure 5 (*P*=0.19, *I*^2^ = 37%), so these few. There is no heterogeneity between the two studies. Next, a fixed-effect model is used to conduct meta-analysis on the imported data, and the combined effect size (OR = 1.79, 95% CI (0.96, 3.35)). The results showed that the CR of the albumin paclitaxel group for breast cancer was higher than that of the docetaxel group (*Z* = 1.83, *P*=0.07), which indicated that the difference was not statistically significant. This result indicates that there is no significant difference between the albumin paclitaxel group and the docetaxel group in the treatment of breast cancer CR.

#### 3.3.3. Partial Response Rate (PR)

In this study, 4 articles reported two paclitaxel PR in treatment of breast cancer patients and extracted data, using RevMan5.3 software to test their heterogeneity, as shown in Figure 6 (*P*=0.57, *I*^2^ = 0%), so there is no heterogeneity among these studies. Next, a fixed effect model was used to conduct meta-analysis of the imported data and the combined effect (OR = 0.88, 95% CI (0.53, 1.47). The results showed that the PR of the paclitaxel group was lower than that of the Western Taxus group (*Z* = 0.49, *P*=0.62), which indicated that the difference was not statistically significant. This result suggested that there was no significant difference between the paclitaxel group and the docetaxel group in the PR treatment of breast cancer.

#### 3.3.4. Neutropenia

In this study, there are two literature reports on the reduction of mesoparticle cells in two types of paclitaxel treatment of breast cancer patients. The data were extracted, and the heterogeneity was tested using RevMan5.3 software, as shown in Figure 7 (*P*=0.20, *I*^2^ = 39%), Therefore, there is no heterogeneity between these several studies, and then the fixed effects model is used to conduct meta-analysis on the imported data and the combined effect size (OR = 0.38, 95% CI (0.16, 0.88)). The results show that the reduction of neutrophils in the albumin paclitaxel group in the treatment of breast cancer was lower than that in the docetaxel group (*Z* = 2.25, *P*=0.02), which indicated that the difference was statistically significant. This result suggested that the albumin paclitaxel group has a lower risk of neutropenia in the treatment of breast cancer than the docetaxel group.

#### 3.3.5. Nausea

In this study, there are 3 literature studies reporting the incidence of nausea in the adverse reactions of two types of paclitaxel treatment in breast cancer patients. The data were extracted, and the heterogeneity was tested using RevMan5.3 software, as shown in Figure 8 (*P*=0.87, *I*^2^ = 0%), so it is concluded that there is no heterogeneity between these studies, and then the fixed effects model is further used to conduct meta-analysis on the imported data and the combined effect size (OR = 0.94, 95% CI (0.51, 1.74)), and the results showed that the incidence of nausea during breast cancer treatment in the albumin paclitaxel group was lower than that in the docetaxel group (*Z* = 0.21, *P*=0.84), which indicated that the difference between the two groups was not statistically significant. This result suggested that there is no significant difference in the incidence of nausea in the treatment of breast cancer between the paclitaxel group and the docetaxel group.

#### 3.3.6. Vomiting

In this study, there are 3 literature reports on the incidence of vomiting of two kinds of adverse reactions of paclitaxel treatment in breast cancer patients. The data were extracted, and the heterogeneity was tested using RevMan5.3 software, as shown in Figure 9 (*P*=0.62, *I*^2^ = 0%), so there is no heterogeneity between these several studies, and then the fixed-effects model is further used to meta-analyze the imported data and the combined effect size (OR = 0.90, 95% CI (0.45, 1.78)). The results showed that the incidence of vomiting in the treatment of breast cancer in the albumin paclitaxel group was lower than that in the docetaxel group (*Z* = 0.34, *P*=0.76), which indicated that the difference shown in the results was not statistically significant. This result shows that there is no significant difference in the incidence of vomiting in the treatment of breast cancer between the albumin paclitaxel group and the docetaxel group.

### 3.4. Publication Bias

Because there are only four articles included in the Meta analysis of this study, the test performance is too low, so the funnel chart analysis is not performed for this.

## 4. Discussion

Breast cancer is a common malignant tumor in gynecology, and its incidence and mortality have long been ranked first among all tumors in women [12]. Breast cancer is mainly due to malignant canceration of breast ductal epithelium or breast acinar epithelial cells. Breast cancer cells are different from normal cells [13–15]. Compared with normal cells, breast cancer cells grow and divide very quickly, and they like to attack normal tissues of the body [16]. At the same time, breast cancer cells are easy to adhere to due to the decreased intercellular adhesion of breast cancer cells. It spreads to other parts through blood circulation and adheres and proliferates in other parts [17, 18]. In this regard, while comparing the efficacy of albumin paclitaxel and docetaxel in the treatment of breast cancer patients, this study also conducted a comparative evaluation of its adverse reactions.

The four articles in this study are all high-quality English literature. The objective of this study is to evaluate the effectiveness of two paclitaxel in the treatment of breast cancer from the aspects of objective effectiveness (ORR), complete remission (CR), partial remission (PR), neutrophils reduction, nausea, and vomiting [19, 20]. The research shows that, in the combined analysis of various outcome indicators, it is found that the heterogeneity of the included studies is small, but most of the differences are not statistically significant, and most of the literature cannot specifically describe whether to use the method of random allocation and allocation concealment. Most studies are affected by the disease and cannot use the blind method [21]. The results of meta-analysis showed that the treatment of breast cancer with paclitaxel group and docetaxel group can reduce the risk of neutrophils in breast cancer patients, which is closely related to the follow-up treatment, but in contrast to objective effective rate (ORR), complete remission (CR), partial remission (PR), nausea, and adverse reactions, There was no significant difference in vomiting between the two groups.

The results of this study show that the use of albumin paclitaxel for clinical treatment can better reduce the incidence of neutropenia in breast cancer patients, which is of great significance for breast cancer patients. However, this study also has some relative limitations, such as the number of included clinical studies is small, and the sample size is small. There is a lack of data support, and the design of clinical studies still needs to be further planned and perfected. This also shows that if you want to get more evidence-based conclusions, a large sample of clinical experimental research and data should be actively carried out and collected. While providing reference for the clinical treatment plan of breast cancer patients, further analysis should also provide evidence-based evidence for the clinical treatment outcome of breast cancer patients. The limitations of this study are as follows. ①The number of clinical studies included is small, and there are no more studies on the safety and efficacy of albumin paclitaxel compared with docetaxel in the treatment of breast cancer patients after surgery. ②The various interventions included in the study are different, the interval between patients' medication is inconsistent, and the selection criteria and types of the patient population are different, so the combined results may have a certain impact. ③Since the number of studies included in the meta-analysis was less than 10, no funnel plot analysis was performed, and there may be publication bias.

## Figures and Tables

**Figure 1:** Flow chart of literature screening.

**Figure 2:** Cochrane bias risk percentage of included literature.

**Figure 3:** Cochrane quality percentage of included literature.

**Figure 4:** Meta analysis of ORR comparison between the two groups.

**Figure 5:** Meta-analysis of PR comparison between the two groups.

**Figure 6:** Meta-analysis of PR comparison between the two groups.

**Figure 7:** Meta-analysis chart of the comparison of neutropenia between the two groups.

**Figure 8:** Meta-analysis of the comparison of nausea between the two groups.

**Figure 9:** Meta-analysis of the comparison of vomiting between the two groups.

**Table 1:** Basic characteristics of included literature.

Included literature	Publication time	Subjects (experimental group and control group)	*P*
Qi et al. [8]	2017	29/38	*P* > 0.05
Sparano et al. [9]	2015	26/30	*P* > 0.05
Gradishar et al. [10]	2012	39/39	*P* > 0.05
Watanabe et al. [11]	2015	21/21	*P* > 0.05

## Data Availability

The simulation experiment data used to support the findings of this study are available from the corresponding author upon request.
